# A Liver Segmentation Method Based on the Fusion of VNet and WGAN

**DOI:** 10.1155/2021/5536903

**Published:** 2021-10-08

**Authors:** Jinlin Ma, Yuanyuan Deng, Ziping Ma, Kaiji Mao, Yong Chen

**Affiliations:** ^1^College of Computer Science and Engineering, North Minzu University, Yinchuan, China 750021; ^2^Key Laboratory of Images & Graphics Intelligent Processing of National Ethnic Affairs Commission, Yinchuan, China 750021; ^3^College of Mathematics and Information, North Minzu University, Yinchuan, China 750021; ^4^Department of Interventional Radiology, General Hospital of Ningxia Medical University, Yinchuan, China 750004

## Abstract

Accurate segmentation of liver images is an essential step in liver disease diagnosis, treatment planning, and prognosis. In recent years, although liver segmentation methods based on 2D convolutional neural networks have achieved good results, there is still a lack of interlayer information that causes severe loss of segmentation accuracy to a certain extent. Meanwhile, making the best of high-level and low-level features more effectively in a 2D segmentation network is a challenging problem. Therefore, we designed and implemented a 2.5-dimensional convolutional neural network, VNet_WGAN, to improve the accuracy of liver segmentation. First, we chose three adjacent layers of a liver model as the input of our network and adopted two convolution kernels in series connection, which can integrate cross-sectional spatial information and interlayer information of liver models. Second, a chain residual pooling module is added to fuse multilevel feature information to optimize the skip connection. Finally, the boundary loss function in the generator is employed to compensate for the lack of marginal pixel accuracy in the Dice loss function. The effectiveness of the proposed method is verified on two datasets, LiTS and CHAOS. The Dice coefficients are 92% and 90%, respectively, which are better than those of the compared segmentation networks. In addition, the experimental results also show that the proposed method can reduce computational consumption while retaining higher segmentation accuracy, which is significant for liver segmentation in practice and provides a favorable reference for clinicians in liver segmentation.

## 1. Introduction

Liver cancer (LC) is a common cancer in clinical practice [1], which poses a great threat to the quality of life of patients and their families. With advanced medical technology, early diagnosis and treatment of liver cancer have increased the possibility of curing liver cancer. Therefore, reliable, quick, and precise liver segmentation algorithms have become a major research hotspot in the industry. Generally, traditional liver segmentation methods, including the active contour model [2], clustering [3], level set [4], graph cut method [5–7], and regional growth [8, 9] method, extracted grayscale, shape, structure, and texture information of medical images to segment the liver manually. The efficiency of these methods is limited to large databases. However, its preprocessing of data is time consuming using these methods. However, deep learning performs better than traditional liver segmentation methods in terms of versatility and efficiency.

Among deep learning networks, FCN [10] and UNet [11] are typical segmentation models used in medical image segmentation methods. Subsequently, many networks were derived from these two networks, for example, UNet++ [12] and H-DenseUNet [13]. In practice, the segmentation performance of these networks is similar to that of traditional segmentation methods. UNet is suitable for small-scale medical image data with a relatively single image structure. However, further work needs to be investigated to improve the segmentation accuracy of UNet. Therefore, some traditional methods combining UNet have been proposed to optimize the performance results, such as the method in [14]. A mean shift clustering algorithm was added to reduce the oversegmentation of the liver. To further improve the accuracy of image enhancement, an image enhancement technique based on a statistical threshold is proposed, which excludes nonliver regions by using the cumulative distribution function (CDF). To improve training and inference speed, the literature [15] combined subpixel convolution [16] with bilinear interpolation [17] in the last layer. However, it is difficult to improve the segmentation accuracy because 2D segmentation networks lack sufficient information between slice layers and model learning. To solve this problem, Wang and Wang [18] used the input layer to segment and process 3D images, including using a certain range of layers as an aid, using multiplane integration, training on the axial, sagittal, and coronal planes, and fusing the final segmentation.

The use of 2D and 3D convolution networks has achieved good performance in liver segmentation. A hybrid method [19] inherited the advantages of 2D and 3D convolutions and ignored their disadvantages to the maximum extent possible. It combined 2D Dense-UNet and 3D Dense-UNet to operate on the region of interest through them and extracted intralayer and interlayer features separately. Thus, the segmentation accuracy was improved to a certain extent.

Generally, without considering the calculation and memory performance, 3D networks can utilize the information between adjacent layers to ensure the continuity of changes between the image masks. The VNet network [20] is a 3D neural network for medical image segmentation. It directly uses 3D convolution operations to process 3D volume data instead of 2D slices, effectively exploiting the 3D data spatial information to ensure that the images are marked.

In summary, compared with the 2D convolutional neural network (CNN), 3D CNNs have a large parameter amount, high video memory occupancy rate, and hardware resource intensive, which has largely restricted its advancement and research.

Although the above models can obtain relatively accurate segmentation results in medical image processing, the difficulties in data acquisition and annotation largely hinder the construction of a sufficiently large dataset. To overcome this problem, conventional image enhancement techniques, such as geometric transformation, can generate new data. However, they are unreliable in detecting biological changes in medical data, which can result in limited segmentation performance improvement. In 2014, Goodfellow et al. [21] proposed a generative adversarial network (GAN) model. It uses unsupervised training methods for training through adversarial learning. The purpose is to estimate the potential distribution of the data samples and generate new data samples. Li et al. [22] used GAN to enhance ocean data for research on the detection of climate anomalies. GAN can also realize the conversion between different modal images, using CycleGAN to convert contrast CT images into noncontrast CT images [23], and convert face sketches into RGB images [24].

As GAN does not need to know the theoretical distribution in advance, it can automatically infer the real dataset, which further expands the size and diversity of the data, provides a new method for data expansion, and alleviates the problem of data demand for intelligent diagnosis. Luc et al. [25] applied GAN to image segmentation for the first time. Generally, the semantic segmentation results often need to be improved using CRF and other postprocessing techniques to obtain more realistic contours. Thus, GAN itself has excellent generation capabilities and can be used to improve the results. However, GAN has drawbacks such as unstable training, disappearing gradients, and mode collapse. Based on these issues, numerous popular architectures have been derived involving conditional GAN (CGAN) [26], DCGAN [27] (deep convolutional GAN), and InfoGAN [28] (Information Maximizing GAN). They have solved the drawbacks of GAN to a certain extent. However, there still are some deficiencies in solving the stability problem during the training process. The emergence of WGAN [29] solves the problem of instability in GAN training. Nevertheless, its network structure is very simple, and only a few improvements have been made on the basis of GAN.

Considering the small amount of medical image data coupled with GPU restrictions, the use of 3D data can cause overfitting problems. Therefore, this paper proposes an improved VNet and 2.5-dimensional convolutional neural network VNet_WGAN to obtain the context information of 3D data to realize end-to-end segmentation of liver images. The main tasks are as follows:

1. By using the stack of slices and their upper and lower adjacent slices as the network input and the segmentation map corresponding to the central slice as the output, two convolution kernels in series are used to fully extract the intralayer and interlayer information to adopt for the 3D liver. While maintaining high segmentation accuracy, spatial characteristics can reduce the memory occupancy rate and the amount of calculation
2. To make full use of the high-level and low-level features of the network, a chain residual pooling module is added to the long-skip connection structure of the VNet network to obtain richer semantic information and effectively improve the accuracy of liver segmentation
3. Introduce the boundary loss function into the basic WGAN generator network to compensate for the lack of consideration of the marginal pixel accuracy of the Dice loss function. Utilizing the composite loss function of boundary and Dice weighted fusion, the segmentation ability of the model is enhanced from the region and the boundary, respectively

## 2. Methodology of This Article

### 2.1. GAN

A GAN is a generative confrontation network composed of a generative model *G* and a discriminant model *D*. It can be expressed as a minimax game problem between *G* and *D*. *G* learns the distribution of a given noise (such as uniform distribution and normal distribution) and synthesizes them. *D* distinguishes whether the training sample comes from a real sample or a generated sample.

GAN uses the concept of adversarial learning to achieve better generation results. Adversary means that the images generated by the generative model *G* will become realer and realer when the discriminative ability of the discriminant model *D* becomes stronger and stronger, which finally reach a balance. The basic structure of the GAN is shown in Figure 1. In Figure 1, *x* is the real data, *D*(*x*) represents the score of the real data after being processed by discriminant model *D*, *z* represents the given random variable, the image *G*(*z*) is generated after being processed by generative model *G*, and *G*(*G*(*z*)) represents the image generated by the generative model *G* after the *D* fraction. The formula is given in Equation (1) as follows:

(1) $$\begin{array}{c} \max_{G}\max_{D}V\left(D,G\right)=E_{x\sim P_{\text{data}}\left(x\right)}\left[\log D\left(x\right)\right]+E_{x\sim P_{z}\left(z\right)}\left[\log\left(1-D\left(G\left(z\right)\right)\right)\right]. \end{array}$$

### 2.2. WGAN

The GAN model has interested many researchers. However, the training of a GAN is difficult compared to an ordinary CNN. The main difficulty is balancing the generator and the discriminator and the lack of appropriate indicators to measure the training effect in the training process. Based on these issues, many popular architectures have been designed based on GAN, such as conditional GAN (CGAN), deep convolutional GAN (DCGAN), and information-maximizing GAN (InfoGAN).

Although these methods can solve some of the current problems of GAN to a certain extent, the process stability problem is not yet solved. WGAN solves the problem of training instability while providing a reliable indicator, the Wasserstein distance, for training. Compared with JS (Jensen-Shannon) and KL (Kullback–Leibler), the Wasserstein distance can naturally measure the discrete distribution and the distance between continuous distributions, which completely avoids the common problems of stable training and gradient disappearance in GAN.

The formula of Wasserstein distance is shown in Equation (2) as follows:

(2) $$\begin{array}{c} \max_{G}\max_{D}V\left(D,G\right)=E_{x\sim P_{\text{data}}\left(x\right)}\left[D\left(x\right)\right]+E_{x\sim P_{z}\left(z\right)}\left[D\left(G\left(z\right)\right)\right]. \end{array}$$

### 2.3. VNet

The VNet network structure involves an encoder and a decoder. The encoder was divided into multiple stages, and each stage had the same resolution. The decoder is a gradual decompression path and can finally obtain an output image of the same size as the original image. VNet inherits the jump connection of the UNet to compensate for information loss in the feature extraction process. In addition, VNet uses the short-circuit connection mechanism of ResNet [30] to add the input and output of each stage to learn the residual function.

Meanwhile, the Dice loss function is used to replace the cross-entropy loss function to improve the sensitivity of the target segmentation area. For example, Zhu et al. [31] added the channel attention mechanism [32] to the VNet network structure to segment various organs in the head and neck image.

Milletari et al. used a VNet network in which the encoder part extracts the liver global features from the input image, and the decoder part generates a full-resolution output. Simultaneously, random nonlinear transformation and histogram matching are used to increase the data in the preprocessing. Although the VNet network provides a reference for processing 3D medical images, the medical image data are mostly small with limited GPU memory, which still results in overfitting and instability of the network in the training process, especially for 3D data.

## 3. Methods

As the WGAN model entirely solves the problem of training instability of GAN, therefore, in the training process, it no longer needs to balance the training level of the generator and the discriminator carefully. Because of this excellent characteristic of WGAN, we employed WGAN as the basic structure of our model and designed an improved VNet as the generator for liver segmentation.

In our network, the discriminant network is a simple CNN network that determines whether the input image is a “fake image” (the result of segmentation) or a “real image” (annotated image) generated by the generator. The entire network framework of the proposed method is illustrated in Figure 2.

In Figure 2, the original three adjacent liver images are used as the input, and the improved VNet is used for segmentation. Then, the mask image and the output image obtained by the generation network of VNet are input to the classification structure, in which true can be distinguished from false, where result 1 denotes true and 0 denotes false.

### 3.1. Generator

Owing to the time cost and the ability of feature extraction, the generator used in our method adopts VNet as the backbone network and modifies the original network in a targeted manner. The input of our network is the relevant slice and its two adjacent upper and lower slices, and the median slice was used as the output result. During the training process, convolution kernels with a size of 1 × 3 × 3 and 3 × 1 × 1 were used to extract the intralayer and interlayer information. This convolution approach is similar to separable deep convolution, which can extract 3D features of medical data without extensive calculations generated by a 3D CNN and shortens the training time. The improved convolution module is shown in Figure 3. In the improved convolution module, two chained residual pooling modules, CRP (chained residual polling) with pooling and convolution operations, are added to the jump connection part of the VNet to make more effective use of high-level and low-level feature information.

The chained pooling operations can considerably increase the receptive field in that edge information can be extracted from high-resolution feature maps, and global information can be extracted by low resolution. Therefore, the classification accuracy of the pixels is further improved.

Meanwhile, the residual structure is beneficial to the inverse spread of the gradient. As can be seen in Figure 4, the module includes two pooling convolution blocks, two residual structures, one activation function, batch normalization, and dropout layers. The network uses a convolution kernel of 1 × 5 × 5, padding 2, and stride 1 to perform pooling operations to ensure that the image size after pooling is consistent with the input image size. The pooling is followed by a convolution operation, and then, the output result is input to the next pooling convolution module. Finally, the two feature maps are merged.

In the network training process, the more complex the network model, the more the features need to be learned, which require more training time and easily lead to overfitting problems. Therefore, this study made slight adjustments to the existing network model.

Specific ways are that batch normalization (BN) is added to normalize the data with different distributions after each revolution. Thus, each layer of data can be transformed into the same distribution.

Therefore, the optimal result of the network model converges more easily, so that the training speed of the network model is accelerated to a great extent.

Adding a dropout layer can solve the scenario in which some features are only useful when other features exist, also enhance the robustness of the neural network, effectively alleviate the overfitting issues, and achieve regularization to a certain extent.

Figure 5 shows the structure of the improved VNet in this study, which retains the characteristics of the encoder-decoder structure. The entire network contains five convolution blocks, four deconvolution blocks, and the last convolution output layer. The encoding path above is divided into five stages, and each stage contains two convolution blocks with the same resolution. Each convolution block is composed of a convolution kernel, normalization, and ReLU activation function, using 32 in turn. These convolution blocks employ 64, 128, 256, and 256 channels of the convolution kernel, with a moving step of 1, to extract the features.

To reduce the memory used in the training process, convolution is used to replace the pooling operation in the downsampling process with a 1 × 3 × 3 convolution kernel and a moving cloth of 2 in length. This pooling operation approach can reduce the image resolution. Moreover, to learn features at each stage, the input and output in each stage are added together to perform short-range residual learning.

Upsampling is performed before decoding using 512 1 × 3 × 3 convolution kernels with a step size of 2 for the deconvolution operation.

The decoder path below is divided into four stages, and each stage has the same resolution. A convolution kernel with a size of 1 × 3 × 3 is used to restore the size of the feature map and expand the low-resolution space.

Through four upsampling operations, an image with the same resolution as the input image is finally obtained. Simultaneously, the original VNet network transforms the results of each stage in the encoder to the input and directly adds it to the input of the corresponding stage in the decoder, retaining some information loss owing to compression.

After a chain residual pooling module consisting of a pooling layer, a convolutional layer, and a residual structure, efficient pooling is performed through different convolution kernels, where the size of the output feature map is consistent with the input. Then, the corresponding stage is added as the input for the next stage. The last convolution layer applies a 1 × 1 × 1 convolution kernel to obtain an image of the same size as the input. The specific network parameter distributions are listed in Table 1.

### 3.2. Discriminator

The network structure of the discriminator used in this approach is shown in Figure 6. The inputs of the discriminator are the output result of the generator and the annotated image of the original image, which are first fused and then input to the CNN network. Finally, the second classifier outputs the output signal of the discriminator.

The discriminator includes one group of conditional pooling blocks, four groups of convolutional blocks, two fully connected layers, and the last two classification layers. A group of convolutional pooling blocks contains two convolutional layers and one maximum pooling layer. Each convolutional layer is composed of a convolution kernel, normalization, and an activation function.

The size of the convolution kernel was 1 × 3 × 3, with a moving distance of 1. A total of 64 convolution operations were used in the 1st convolutional block and 2nd conditional block. In the pool process, we choose a 1 × 2 × 2 convolution kernel with a moving distance of 1. In the 3rd and 4th convolution blocks, there are 32 convolution kernels where the size of each convolution kernel is 1 × 3 × 3 with a moving distance of 1. The output of the 4th convolution block was used as the input of the fully connected layer.

### 3.3. Loss Function

The loss function of our method in this paper is composed of the loss function of the generator and the discriminator.

The generator was based on an improved VNet segmentation network. The objective function, Dice loss, was proposed in the VNet network. It can balance background and background information well and is a commonly used loss function in the field of medical image segmentation.

Dice loss is very similar to the Dice coefficient and is used to evaluate the similarity between two regions. The calculation formula of Dice loss is shown in formula (3), where *A* represents the set of all predicted foreground pixels and *B* represents the set of real foreground pixels.

(3) $$\begin{array}{c} L_{\text{Dice}}=1-\frac{2\;|\;A\cap B\;|\;}{\;|\;A\;|\;+\;|\;B\;|\;}=\frac{\;|\;A\;|\;-\;|\;A\cap B\;|\;+\;|\;B\;|\;-\;|\;A\cap B\;|\;}{\;|\;A\;|\;+\;|\;B\;|\;}. \end{array}$$

Dice loss focuses more on the similarity of regions and ignores spatial information, such as missegmentation sections far away from the label region. Therefore, to minimize the distance between the segmentation boundary and the label boundary, a synthetic function of Dice loss and boundary loss [33] is proposed. In this synthetic function, boundary loss controls the degree of network loss by the edge matching degree.

The synthetic function evaluates only pixels on the boundary. The boundary loss value equals 0 when the pixels on the boundary are entirely consistent with the boundary of the ground truth, whereas it is evaluated by its distance from the boundary when the boundary does not coincide with the real result. The experimental results in this study show that the synthetic loss function is the weighted fusion of Dice loss and boundary loss. Among them, one controls the area and the other controls the boundary, which can achieve better segmentation performance.

In practice, the Dice loss score was very high at the beginning of training. As the training progresses, the proportion of boundary loss increases, which illustrates that accuracy of the boundary gets more attention in the later stages of the training with enhanced boundary detail information being processed. Therefore, we exploit this idea and apply it to the task of liver image segmentation.

Figure 7 shows the relationship between the parameters in the boundary loss formula, where *∂G* represents the boundary of the real segmentation area, *∂S* represents the boundary of the segmentation area output by the network, *p*, *y∂S*(*p*) represent the connection points of the real and predicted results, and Δ*S* represents the area between the two contour lines and *D*_*G*_. To calculate the distance Dist(*∂G*, *∂S*) between the boundaries of the two regions in a differential way, boundary loss uses a split on the boundary to alleviate the difficulties caused by unbalanced segmentation instead of an unbalanced integration of the regions. The boundary loss formula is as follows:

(4) $$\begin{array}{c} L_{BD}=\text{Dist}=\int_{\partial G}{\left|\left|q\partial S\left(p\right)-p\right|\right|}^{2}dp\approx 2\int_{\Delta S}D_{G}\left(p\right)dp=2\left(\int_{\Omega }\phi_{G}\left(p\right)s\left(P\right)dp-\int_{\Omega }\phi_{G}\left(p\right)g\left(P\right)dp\right),\\ D_{G}\left(p\right)=\left|\left|p-Z_{\partial G}\left(p\right)\right|\right|, \end{array}$$

where *D*_*G*_(*p*) represents the distance from the real result, *s*(*p*) and *g*(*p*) are quadratic index functions, and *ϕ*_*G*_ is the boundary level set; if *q* ∈ *G*, *ϕ*_*G*_ = −*D*_*G*_(*q*), otherwise *ϕ*_*G*_ = −*D*_*G*_(*p*), *s*_*θ*_(*p*) is the softmax probability output of the network. The final boundary loss function is

(5) $$\begin{array}{c} L_{BD}=\int_{\Omega }\phi_{G}\left(p\right)s_{\theta }\left(p\right)dp. \end{array}$$

In a sense, both Dice loss and boundary loss minimize the false overlap parts between the segmentation result and the marked result. For Dice loss, the segmentation mismatch is weighted by the sum of the number of foreground pixels in the segmentation and the number of pixels in the real result.

Boundary loss is weighted only by the distance conversion of the real result. The calculation formula of the compound loss function used in this study is 7, where *α* is the weight parameter of the balance loss, and the parameter selected in the experiment was 0.1.

(6) $$\begin{array}{c} L=\alpha *L_{\text{Dice}}+\left(1-\alpha \right)*L_{BD}. \end{array}$$

Loss function of discriminator. Because the discriminator is based on the same network structure as WGAN, the Wasserstein distance is used as the loss function, which is given by

(7) $$\begin{array}{c} L_{D}=\min_{G}\max_{D}E_{x\sim P_{r}\left(x\right)}\left[D\left(x\right)\right]-E_{z\sim P_{z}\left(z\right)}\left[D\left(G\left(z\right)\right)\right]. \end{array}$$

## 4. Experiments

### 4.1. Experimental Data

To evaluate the actual effect of the method in the application of liver segmentation, experiments were carried out on the LiTS and CHAOS datasets. The LiTS dataset includes 130 contrast-enhanced 3D abdominal CT images from six different clinical sites in nii format. The original CT data were named by volume-∗.nii, and the ground-truth image is named by segmentation-∗. nii.

It contains 130 sets of training data and 70 sets of test data, of which 70 sets of test data were unlabeled. The CT image containing 908 lesions was provided by reference annotations of the liver and tumor made by experienced radiologists.

The dataset has significant differences in image quality, spatial resolution, and vision. The in-plane resolution is 0.6 × 0.6 ~ 1.0 × 1.0 mm, and the slice thickness (interlayer spacing) is 0.45~6.0 mm. All scanning axial slice sizes were fixed at 512 × 512 pixels, with the number of slices per scan ranging from 42 to 1026.  Figure 8 shows the visualization results of liver tumor images in the LiTS dataset.

The CHAOS dataset is a dataset with multiorgan, multimodal segmentation, which includes images and labeled images of the spleen, liver, left kidney, and right kidney.

The datasets have two modal databases: CT and MRI. In the two databases, each dataset with .dcm format corresponds to an image of a single patient, and each image corresponds to a slice.

The dataset was provided by the PACS of the DEU Hospital. In this study, we used an MRI database, which contains two modalities, T1-DUAL and T2-SPIR, each with 40 datasets. T1-DUAL is divided into two categories: InPhase and OutPhase.

In this study, T1-DUAL/InPhase was selected as the dataset. The rule of naming images is the same as that used to annotate images in this dataset. Thus, processing is relatively simple. The training and test sets were divided into 20 cases. The MRI image can generate 12-bit DICOM images with a resolution of 256 × 256 and a number of slices between 26 and 50. Because the test set does not provide annotated images, this study uses 20 labeled cases to redivide them into training set and test set, of which 16 cases were used as the training set, and four cases were used as the test set. One of the processed liver images and the labeled image of the liver are illustrated in Figures 9(a) and 9(b), respectively.

### 4.2. Experimental Setting

The experimental environment was as follows: the computer operating system was Windows10, the main hardware devices were two NVIDIA GTX1080 GPUs, the memory was 8 GB, and the development tools were Python and TensorFlow.

### 4.3. Evaluation Index

In the experiment, the accuracy and Dice similarity coefficient (DSC) were used to quantitatively measure the performance of image segmentation algorithms in medical image segmentation tasks. The accuracy represents the proportion of correct data to the overall data. The calculation formula is as follows:

(8) $$\begin{array}{c} \text{Accuracy}=\frac{\text{TP}+\text{TN}}{\text{TP}+\text{TN}+\text{FP}+\text{FN}}, \end{array}$$

where *P* (Positive) and *N* (Negative) represent the prediction results of the model, *T* (True) and *F* (False) are used to judge whether the results of the model are correct, and FP (False Positive), FN (False Negative), TP (True Positive), and TN (True Negative) represent false positive, false negative cases, true cases, and true negative cases, respectively.

Figure 10 shows the correlations between the above symbols. In Figure 10, *A* denotes the image containing the theoretical segmentation result that is used for comparison with the resulting image, and *B* is the predicted segmentation result.

The Dice similarity coefficient (DSC) is mainly used to evaluate the similarity of the distance between the segmentation result and the marker result. Its value ranges from 0 to 1, where 0 means that the experimental segmentation result deviates from the marking result seriously, while 1 demonstrates that the experimental segmentation results completely overlap with the labeled results; that is, the higher the evaluation results, the higher the accuracy of the segmentation. The formula for calculating Dice is as follows:

(9) $$\begin{array}{c} \text{Dice}=\frac{2\;|\;A\cap B\;|\;}{\;|\;A\;|\;+\;|\;B\;|\;}=\frac{2\text{TP}}{2\text{TP}+\text{FP}+\text{FN}}. \end{array}$$

## 5. Results

### 5.1. Method Comparison Test

In this section, experiments are designed to verify the effectiveness of the proposed algorithm VNet_WGAN, which is compatible with 3D UNet, 2.5DVNet, UNet, Attention [34], CycleGAN [35], and DenseNet, which are suitable for various medical image segmentation tasks. The results of the comparative experiments are presented in Table 2. It can be concluded from Table 2 that compared with other algorithms, VNet_WGAN has a certain improvement in accuracy and Dice coefficient, particularly in the Dice coefficient. Compared with 3D UNet, although the Dice value of VNet_WGAN is not significantly different, it also increases by at least 1%. Compared with 2D segmentation networks including UNet, Attention, CycleGAN, and DenseNet, the accuracy and Dice score of VNet_WGAN were significantly improved. For example, CycleGAN grew by 8% and 3%, respectively. Therefore, VNet_WGAN is appropriate and efficient for solving the problem of liver segmentation.

### 5.2. Loss Function Comparison Test

To evaluate the effect of the loss function of VNet_WGAN designed in this study on liver segmentation, a comparative ablation experiment was performed on the LITS dataset, using the five most common loss functions in liver segmentation: IoU loss, cross-entropy loss, Dice loss, boundary loss, and the compound loss function used in this study. Moreover, VNet_WGAN was designed in this study, and the improved 2.5D VNet model was used as the comparison model. All experimental training configurations were identical. The IoU loss is the loss function calculated by IoU to obtain the gradient for regression. Cross-entry loss refers to the difference between the two probability distributions. The amount of information is inversely proportional to the probability of the occurrence of information. Dice loss is proposed in the original VNet network and is an ensemble similarity measurement function that is used to calculate the similarity between two samples. The composite loss function is a loss function that combines the boundaries and regions. The performances of these five loss functions in the two network models are listed in Tables 3 and 4, respectively.

From Tables 3 and 4, it can be observed that with the loss function of this study, the improved 2.5D VNet model achieves an accuracy of 96% in the liver segmentation task and a Dice of 89%. In the fusion model of VNet_WGAN, the accuracy was 94%, and the Dice was 92%. In the same network model, the composite loss function has little difference in accuracy, but it performs very well in terms of Dice, which is 1% higher than Dice loss. In the same dataset and the same loss function, the method in this study improves in terms of Dice by 3%.

Through the ablation experiment and the above analysis, it is shown that our composite loss function, the weighted fusion of boundary loss and Dice loss, can improve the accuracy and precision of the segmentation results, indicating that the design of our composite loss function has a certain guiding significance for the extraction of key features of the network. This demonstrates that our composite loss function can extract detailed information of features effectively and accurately, which plays an important role in solving the poor performance of image segmentation methods.

### 5.3. Visualization of the Experimental Results

To observe the segmentation effect more intuitively, in this section, we conduct a qualitative analysis of the models covering the segmentation algorithm fused with VNet and WGAN and the 3D VNet segmentation algorithm on the LITS dataset.  Figure 11 shows the visual segmentation results of the two segmentation algorithms. In the experiment, six layers of images were selected for comparison. Lines 1-4 in the figure are the original images, the image annotated by the clinician manually, the 3D VNet segmentation results, and the segmentation results of the fusion of VNet_WGAN.

From the segmentation results in the figure, it can be seen that the segmentation algorithm of 3D VNet and the fusion of VNet and WGAN do not perform very well in the early and late regions of the liver, whereas in the midterm, the prediction results and the annotation results are extremely coincident. In addition, it is also illustrated that the segmentation algorithm fused by VNet and WGAN has more accurate segmentation results than 3D VNet, which is clearly conspicuous on the boundary contour, as can be seen from the 3-5 columns of Figure 11. Even in the later stage, when the segmentation effect is relatively poor, the segmentation algorithm fused with VNet and WGAN still exhibits good performance. As shown in the sixth column of Figure 11, the segmentation effect of the 3D VNet is somewhat different from the annotation outcome. This proves that the segmentation effect of the algorithm in this study is more refined and closer to the results of expert manual segmentation.

## 6. Conclusion

In this study, we used the VNet_WGAN network to automatically segment the liver to overcome current difficulties in liver segmentation tasks. The algorithm solves the lack of interlayer information of the data in the 2D segmentation network, adopts three adjacent slices as input, and uses two convolution kernels to enhance the context information of the 3D data. Therefore, our method effectively improved the segmentation accuracy. In terms of network structure design, the link residual pooling is introduced into the VNet, the skip connection part is improved, and the high-level feature information and low-level feature information are efficiently fused in the feature extraction part. Moreover, to optimize the model's ability to learn features during the training process, the composite loss function of the weighted fusion of boundary loss and Dice loss is used as the loss function of the generator to ensure clearer edge and texture information. In this study, experiments were conducted on two datasets, LiTS and CHAOS, to verify the effectiveness and generalization of the VNet_WGAN segmentation algorithm. Experimental results show that compared with other segmentation algorithms, the proposed method improves the Dice value by at least 3% while a high segmentation accuracy is maintained by reducing memory usage and calculation amount. This provides a powerful reference for clinicians to perform liver segmentation.

However, the scope of application of the algorithm has certain limitations, in which the loss function part is suitable for other medical image processing tasks, such as lung nodule detection and brain tumor segmentation. In the follow-up work, further refinement and segmentation of the tumor on this basis is the main aim of research in the future.

## Figures and Tables

**Figure 1:** Basic structure of GAN.

**Figure 2:** Structure diagram of VNet_WGAN.

**Figure 3:** Improved convolution module.

**Figure 4:** Chain residual pooling module.

**Figure 5:** Structure diagram of liver segmentation generator.

**Figure 6:** Structure of liver segmentation discriminant.

**Figure 7:** Parameter relationship.

**Figure 8:** Example of liver tumor images in the LiTS dataset.

**Figure 9:** Example of liver images in the CHAOS dataset.

**Figure 10:** Concepts related to evaluation indicators.

**Figure 11:** Comparison of prediction results.

**Table 1:** Network parameter.

Network layer	Number of feature maps	Feature map size/pixels	Number of participants/each
Convolutional layer 1	32	128 × 128 × 128	896
Convolutional layer 2	32	64 × 64 × 64	27680
Convolutional layer 3	64	32 × 32 × 32	110656
Convolutional layer 4	128	16 × 16 × 16	442496
Convolutional layer 5	256	8 × 8 × 8	1769728
Convolutional layer 6	256	4 × 4 × 4	1769728
Deconvolution 1	512	8 × 8 × 8	3539456
Convolutional layer 7	256	8 × 8 × 8	5308672
Deconvolution 2	256	8 × 8 × 8	1769728
Convolutional layer 8	128	16 × 16 × 16	1327232
Deconvolution 3	128	32 × 32 × 32	442496
Convolutional layer 9	64	32 × 32 × 32	110656
Deconvolution 4	64	64 × 64 × 64	82976
Convolutional layer 10	32	64 × 64 × 64	82976
Deconvolution 5	64	64 × 64 × 64	82976
Convolutional layer 11	32	128 × 128 × 128	27680
Convolutional layer 12	32	128 × 128 × 128	55328
Fully connected layer	1	128 × 128 × 128	33
Total	-	-	22482273

Note: “-” means no data.

**Table 2:** The experimental results of different methods were compared.

Comparison method	Dataset	Accuracy	Dice
3D UNet	LiTS	0.98	0.91
3D UNet	CHAOS	0.96	0.89
Improved 2.5D VNet	LiTS	0.96	0.89
3D VNet	LiTS	0.95	0.90
2.5D UNet	LiTS	—	0.77
Attention [34]	LiTS	—	0.76
CycleGAN [35]	LiTS	0.86	0.89
DenseNet	LiTS	—	0.91
Ours (VNet_WGAN)	LiTS	0.94	0.92
Ours (VNet_WGAN)	CHAOS	0.94	0.90

Note: “-” means no data.

**Table 3:** Comparison of segmentation effects of different loss functions in the 2.5D VNet model.

Loss function	Accuracy	Dice
IoU loss	0.96	0.80
Cross-entropy loss	0.95	0.84
Dice loss	0.96	0.88
Boundary loss	**0.97**	0.83
Dice loss+boundary loss (ours)	0.96	**0.89**

Note: the bold font is the optimal value for each column.

**Table 4:** Comparison of segmentation effects of different loss functions in VNet and WGAN fusion models (ours).

Loss function	Accuracy	Dice
IoU loss	0.93	0.86
Cross-entropy loss	**0.95**	0.89
Dice loss	0.94	0.91
Boundary loss	0.92	0.88
Dice loss+boundary loss (ours)	0.94	**0.92**

Note: the bold font is the optimal value for each column.

## Data Availability

Data used in this paper's preparation was obtained from LiTS dataset (https://academictorrents.com/details/27772adef6f563a1ecc0ae19a528b956e6c803ce) and CHAOS dataset (https://chaos.grand-challenge.org/Download/).
